The article "Optimal Cellular Microscopic Pattern Recognizer- (OCMPR-) Based Wireless Detection Network for Efficiently Leveraging the Parallel Distributed Processing Capabilities" was retracted in 2023. Reasons: signs of a paper mill; compromised peer review; unreliable results or conclusions.

# Optimal Cellular Microscopic Pattern Recognizer- (OCMPR-) Based Wireless Detection Network for Efficiently Leveraging the Parallel Distributed Processing Capabilities

**DOI:** 10.1155/2022/5875260

**Published:** 2022-08-06

**Authors:** D. Kaleeswaran, R. Kavitha

**Affiliations:** ^1^Department of Information Technology, Rathinam Technical Campus, Eachanari, Coimbatore, Tamilnadu, India; ^2^Velammal College of Engineering and Technology, Madurai, Tamilnadu, India

## Abstract

Recognizing patterns associated with particular events enables the detection of specific critical changes in the events. Due to the resource constraints inherent in WSNs, pattern recognition is highly dependent on the complexity of the computation, the number of iterations, and the requirements for node training. Iterative learning is frequently used in computer-based computer vision. As a result, these methods are in conflict with the perfectly alright architecture of the WSN. The proposed technique, Optimal Cellular Microscopic Pattern Recognizer (OCMPR), enables the detection of macroscale events in WSN. Using the distributed system computational resources of WSNs, the approach reduces calculations for conserving energy and improves recognition. The method generates promising results by combining a well-known optimization technique (the genetic algorithm) with CMPR. This approach addresses the resource-constrained WSN's real-time mission-critical application needs. Global and quick recognition is achieved by dispersing processing over a network's nodes, allowing for loosely connected communication. The results demonstrate the suggested scheme's versatility.

## 1. Introduction

To detect a single or a group of related events, a network analyses sensory data. Consider structural health monitoring. Install a WSN on the Golden Gate Bridge to collect and analyse vibrations. The same field uses multiscale WSN to detect SHM damage [1]. Another researcher used sensor networks to monitor and detect elderly behaviour. These apps must be able to detect and report accurately in noisy environments [2]. Recognize event-related patterns to detect events. WSN pattern recognition is resource intensive due to computation complexity, iterations, and node training. Computers usually use iterative machine learning. These methods clash with the WSN's highly distributed architecture [3].

This article introduces the Optimal Cellular Microscopic Pattern Recognizer (OCMPR) as a novel computational scheme for resource-constrained WSNs. [4]. Global and rapid recognition is achieved with minimal computational overhead thanks to the proposed scheme's distributed computation and loosely coupled communication. This method solves optimization problems using a genetic algorithm [5].

WSNs collect environmental data through the use of thresholds, statistics, syntactical and associative memories, and graph neurons. Threshold-based pattern recognition is the most basic and widely used WSN pattern recognition technique. These sensors have a single threshold or a set of thresholds. The desired pattern is discovered when a sensor's reading reaches a threshold. Chen et al. [6] created a model that calculates thresholds based on average sensor signal measurements. An alarm is triggered in the event of a threshold violation. The node transmits a DETECT signal to the base station. Simple, light-weight thresholds may exist. These techniques are ineffective against noisy patterns and may result in false alarms [7].

In statistical pattern recognition algorithms, the probability of observing a pattern is used. Assumptions: recognition decisions are made in probabilistic terms, and we are aware of the frequency with which certain events occur [8]. Pattern recognizer must evaluate the model's significance and success probability. Additionally, large-scale and centralized computing resources will be required.

The syntactic model defines subpattern and pattern relationships. It assumes that letters form words, which then form sentences. The model takes syntactic constraints into account when describing the relationships (rules) between subpatterns and primitives that describe patterns [9]. This study examines things using a variety of well-known methods. There are numerous techniques available, including neural networks, tree grammars, and transformations [10]. Syntactic PR is advantageous when a suitable statistical method for deciphering complex patterns is unavailable. On the other hand, developing grammars and recognizer (recognition) is challenging, even more so in the presence of noise [11].

Associative memory, according to Haihong (Zhang) and colleagues, can be used to recognize high-performance patterns (AM). Hopfield [12, 13] demonstrates how AM works by utilizing synaptic weights. The Hopfield network contains numerous connections and dependencies between its nodes. By implementing this method in WSN, the number, size, and complexity of messages sent into and out of the network will increase. Additionally, because the synaptic connections between nodes are established in advance, the system is incompatible with real-time applications. Morphological associative memories (MAM) are used for one-shot learning and pattern recognition in noisy environments [14, 15]. They accomplish this by establishing maximum and minimum matrices. On the other hand, this WSN scheme has two significant flaws. MAM is fundamentally a network. Second, because MAM's calculations are based on global network communication, the length of the learning cycle is difficult to predict. Layers are used extensively in convolutional neural networks to further simplify their operations [16, 17]. It is a system of rules that requires extensive practice. Thus, many connections are required but only a few are used. Yao et al. use SVM to find patterns [18]. By contrast, SVM prefers to maintain a distinct set of pattern representation vectors. As a result, communication and computation are distributed throughout the network. SVM also requires a kernel function to build a dense network [16].

WSNs have been employed as control systems and navigation guidance brains for robots. The work includes examples of such uses. Their hybrid solution uses static sensors to detect events and mobile sensors to steer them to potentially dangerous places on a map. We show how to find obstacles on a map and find a collision-free path between two spots. Pattern recognition and event detection can help robot navigation. A wireless sensor network's pattern recognition detects a pattern. Control systems and robot navigation applications rely on accurate pattern recognition. This is an example of effective detection. WSN resource constraints will impact certain procedures, which have unique requirements. Pattern detection in WSNs necessitates loosely connected connectivity, light-weight computation, memory and resource scalability, and addressing pattern variance. WSN pattern recognition uses threshold-based, closest neighbour, fuzzy logic, and neural network pattern recognition. Several of these techniques necessitate complex computations or communications. Others completely overlook pattern variation. Pattern recognition with variance is necessary for robot guidance.

GA has contributed in the development of robot control systems. Problem size and GA time complexity have an exponential connection, which makes GA challenging to use. How to improve GA performance has been extensively studied. Parameter tweaking, parallel GA, hybrid GA, and more methods exist. Time complexity of GA system improvements is not always predictable. In some cases, reusing previously solved problems can help GA. With GA seeding, the ideal solution is reached in fewer generations. But he noticed that running seeded GA takes nearly as long as running GA with a random beginning population. We hypothesised that exposing a GA to good initial solutions would speed convergence to a good solution (in comparison to a randomly initialised GA). In the same number of generations, a better solution than the GA can be found. First, the GA is run for the provided problem space and then for similar problem spaces. The injected solutions are only partially viable. Otherwise, the GA is starved. A problem space solution should also be generic enough to apply to a wide range of challenges. These requirements demand comparable problem spaces. Pattern recognition is necessary to find solutions. The robot was guided by a scalable AM method capable of effective pattern recognition in wireless sensor networks. In a nutshell, the AM's responsibility was to keep track of previously addressed issues and to resolve them efficiently. Graph Neuron (GN) and Hierarchal Graph Neuron (HGN) are pattern recognition algorithms for wireless sensor networks (WSNs). GN AM distributed fully parallel over fine-grained WSN. Only other GN nodes can communicate with each other. This allows for decentralised learning. These features make GN a good choice for WSN pattern recognition. A bias array memory structure is used by each node to hold the input pattern. Each input pattern is decomposed by the GN array. The GN nodes are activated for each *p* (value, position). Its neighbours dictate its value and position (i.e., previous and next). During memorisation, a node memorises its own and neighbouring value combinations. It will search the bias array for a recall combination. A recall is raised if the combination is in the node's bias array. Each neuron's limited perspective has an effect on the accuracy of GN recognition. As a result, there is crosstalk. If a GN network memorises the patterns ABCDF and FBCDE, the pattern ABCDE will be incorrectly recalled. In Hierarchal Graph Neuron, the crosstalk problem is solved by viewing the incoming pattern through a pyramidal framework (HGN). Distributed HGN reduces the learning cycle and complexity of HGN (DHGN). However, for larger and more complex patterns, the size of HGN and DHGN networks can still grow significantly. We demonstrated the initial version of our Cellular Microscopic Pattern Recognizer (CMPR), a technique similar to HGN but with fewer nodes and no crosstalk. GN, HGN, DHGN, and CMPR all have the ability to analyse distorted patterns. These schemes, on the other hand, are oriented around template matching and ignore pattern dilation, translation, and rotation. The pattern recognition scheme described in this article is highly efficient because it makes use of WSN.

Another option proposed was autonomous robot navigation using GA. This strategy assumes the robot is led by sensors or GPS. It uses GA to generate a collision-free path from the map's top left corner to the bottom right corner. It does so by using two GA chromosomal switching sites. At these points, the robot's direction changes. This method was chosen for robot guiding because it can deal with complex sensory data streams. The algorithmically independent pattern recognition AM given here can be integrated with any other GA issue. The proposed pattern recognition system for WSNs is described next.

Graph Neuron (GN) is a technique for tiny WSN AM. They can only communicate with other GN nodes and are only loosely linked. This allows for decentralised, lightweight one-time learning. So GN is ideal for WSN pattern recognition. A bias array memory structure is created by each node. The pairings of *p* is combination of (value, position). The GN array automatically decomposes each input pattern. The input pattern activates the GN nodes for each *p* pair (value, position). Similarly, each activated node trades value and position information with its neighbours. A node's memory holds its own and other nodes' values. Find a recall match in the bias array. If it finds the bias array, it triggers a recall vote. This is a vote for your node. It remembers the pattern if all neurons respond positively [19].  Figure 1 shows a four-position GN array with ABBA pattern storage and inter-GN communication. A and B are the two options. Because each neuron only sees its immediate surroundings, as a result, GN's vision is impaired. Thus, cross-talk happens. Assume the GN network remembers the patterns ABCDE and FBCDEF. The network will keep the ABCDE but not the ACDE. HGN eliminates cross-talk by building a pyramidal framework that magnifies the incoming pattern [15]. The learning cycle for distributed HGN (DHGN) is shortened [20], not so with DHGN networks. Larger and more complex patterns can be fairly enormous. This article will introduce you to CMPR, a straightforward pattern recognition technique that works well with wireless sensor networks. The WSN's node count is reduced, but the GN's pattern recognition accuracy and one-shot learning capability are maintained. This eliminates a few of the drawbacks associated with other schemes. The following section will go into greater detail about the proposed scheme. A technique called confocal microscopy was used for the detection of microscopic patterns in cells [17].

The classical construction of network topologies provides the way where they use battery to operate and are under continuous monitoring; reports are generated for the phenomenon activities to the node which the central node is called sink node for analysis reasons. WSNs are employed in various vital applications like military and medical field [21]. Though the WSN plays major role in the crisis management, it also suffers some drawbacks like node deployment issue, dependability, energy utilization, and fault tolerance, in order have good communication on continues life time of network in energy efficient, storage, and transmission abilities [22].

The nodes in the WSN show *n* to 1 communication to a single sink which is static leads to the hole in the occurrence nearer to the sink. The balancing of the node helps the consumption of energy and also the link problematical region to isolated segments of the networks which it holds by the sink mobilization. For making the network tolerable, the production of the routing techniques and clustering methods are evolved. Orbital swarming techniques are used in the European space agency (ESA) for self-gathering and interferometer.

Sink mobility in the senor node field is very essential in all applications in real-time environment like battlefield, and natural calamities where the rescuer are fully supported to the find any survivor exist with PDA. The sensor nodes are employed at various different points at required junctions in Intelligent Transport system (ITS) like parking, land sliding prone area which provides premonition to the mobile sink well before to catastrophe event. The lifetime of the networks is by exploiting the mobility of the sink by solving energy hole issue. The sink continuous keeps on changing its location which make topology dynamic. The latest and the recent location of the sink node are monitored to match it with the dynamically changing network topology for maintaining data delivery efficiency. The data propagation protocols show how the retransmission and collision caused by periodic flooding in the sensor field by frequent topological updates. To eradicate the energy meager to the nodes in the field by frequent sink mobility update should be minimized which leads to the energy saver. To minimize the cost of communication the sensor nodes choosing new en route for mobile sink, the virtual infrastructure is superimposed by physical network which is the best method.

Based on the number of neurons in each track, the CMPR network is divided into tracks. Each neuron position contains the same number of nodes as values. If each neuron position contains two nodes, a pattern consisting of nine nodes and two values is produced (i.e., 0 and 1). In the innermost track, only one neuron position, referred to as the “core position” or “core node,” should exist. The goal, it is believed, is to seize control of the entire network. Proceed to the next track with an odd number of locations, beginning at the network's core, in order to establish the tracks' structure. The first position (position 1) in Figure 2 contains two nodes and serves as the network's core. The network's outer track consists of the next three positions (positions 2, 3, and 4), while the outermost track consists of five neuron positions. This is the way a network works. Each neuron receives a segment of a pattern, communicates with its own inner nodes, and exchanges data with other nodes. When a pattern such as 110001001 is displayed to a network, the values 1,1,0,0,0 are displayed. When the pattern 110001001 is displayed, the network will see the values 1 and 1. Each node in each location will behave according to the value assigned to it. If both the node's value and the pattern it receives are 0, the node is activated. This indicates that the node has begun communication with its peers. If this does not occur, the plan will fail. It communicates with other nodes on the same track to deduce the incoming pattern. To report the results of calculations, the active node in position 5 in Figure 2 will communicate with the active nodes in positions 2, 3, and 4.

The incoming pattern is made up of various pattern components. In order to remember the pattern, the node saves the combinations and assigns them a number. The index numbers represent distinct patterns and ascend in order. For example, memorise 001 first. If this is the case, the node will remember the combination and associate it with the number one. The node will assign a new number to the following combination: 011: 2. It is not kept track of whether an existing pattern combination has an index number. Rather than that, the node reports on them using the index number. Utilize the following formula to memorise the index number:

(1) $$\begin{array}{c} N_{k}=\left\{\begin{array}{cc} {SI}_{k}+1, & \text{if no match found}\\ P_{k}, & \text{if a match found} \end{array}\right\}, \end{array}$$

where *N*_*k*_ is the index of the node's output *k*, *SI*_*k*_ is the number of node-stored index *k*, and *P*_*k*_ is the index number for a pattern combination in node *i*'s memory. To recall a pattern, a node examines its memory for a match. If the pattern combinations are old, the node sends index 0. To the right is a schematic showing the index number and recall procedure.

(2) $$\begin{array}{c} N_{k}=\left\{\begin{array}{cc} 0, & \text{if no match found}\\ P_{k}, & \text{if a match found} \end{array}\right\}. \end{array}$$

Because each CMPR position can receive a piece of the pattern, no additional GN nodes are required. Reporting to inner nodes provides a larger view. As a result, the network's size does not match the patterns. A CMPR network has the same physical dimensions as a single-layer GN (but the accuracy of a multilayered HGN). Odd nodes in CMPR: in order to implement the CMPR network design, the following pattern size ceiling must be met:

*N*_TRKS_=$\left\lceil \sqrt{a}\right\rceil .$

To support a pattern of size an, a CMPR network needs to support *N*_TRKS_. As a result, padding is required for certain pattern sizes. To determine the number of padding positions, *N*_PAD_ = (*N*_TKRS_)^2^ − *a*. *N*_PAD_ specifies the number of padding positions. As a result, the following formula can be used to determine the size of the CMPR network, including padding nodes $N\left(a\right)=\text{v}.{\left(\left\lceil \sqrt{a}\right\rceil \right)}^{2}$.

### 1.1. Scheme of Communication

The CMPR Stimulation and Interpreter module sends and receives patterns (S&I). A network entity can execute S&I (i.e., base station). The CMPR communication stages are as follows:

1. Each GN position in the network receives a small portion (pair) of the pattern. The command is to commit the pattern to memory
2. When activated, GNs send messages to adjacent nodes on the same track containing their positions and values
3. Active GNs inspect assisting nodes and S&I for bias array entries. The active GN searches the bias array pattern for the index and returns 0. Each inner GN ignores two nodes. The remaining active node's index numbers will be sent to two neighbouring nodes. Neglected nodes will only talk to their most recent GN. So no more crosstalk
4. This is a fundamental GN number. The S&I saves the index number for each input pattern for memory purposes. That is the pattern of recall. The communication between the GN and the inner track is depicted in Figure 2(c). Neglected GNs communicate directly with nonneglected GNs, while nonneglected GNs communicate with neglected GNs indirectly. GNs on the outer track will receive S&I (current), predecessor node, and successor node

### 1.2. The Complexity of the CMPR Scheme

It is possible to estimate a learning cycle's length by counting tracks, bias array entries, and the time it takes to search a bias array entry. Utilize the following equation to determine the time required for all nodes on the same track to exchange information.

(3) $$\begin{array}{c} T_{1}=2\times \left(N_{\text{TRKS}}-1\right)\times \left(T_{\text{SNT}}+{\text{T}}_{\text{OVRHD}}\right). \end{array}$$

*T*_1_ is omitted from the equation because there are no adjacent nodes at the core node. An array's size affects how long it takes to discover a match. Calculation times are equal to the highest single-node computation times because all nodes in a track compute simultaneously. The overall time depends on tracks rather than nodes.

(4) $$\begin{array}{c} T_{2}=T_{\text{BIAS}}\times N_{\text{ENTRIES}}\times N_{\text{TRKS}}. \end{array}$$

The total reporting time is determined by the number of reporting messages sent between nodes. A node can only send three messages to an inner track node at once. It communicates with the inner and neighbouring nodes when assigned to an inner node. This rule excludes the inner and outermost tracks. Due to the lack of adjacent nodes, the outer track can only report one message per node. Also, all reporting messages are sent concurrently in each track.

(5) $$\begin{array}{c} T_{3}=\left(3\times \left(N_{\text{TRKS}}-2\right)+1\right)\times \left(T_{\text{SNT}}+T_{\text{OVRHD}}\right). \end{array}$$

The sum of the three times *T*_1_, *T*_2_, and *T*_3_ equals the total learning and recall cycle. As a result, the total time can be calculated as shown:

(6) $$\begin{array}{c} T_{\text{TOTAL}}=5\times \left(N_{\text{TRKS}}-7\right)\times \left(T_{\text{SNT}}+T_{\text{OVRHD}}\right)+T_{\text{BIAS}}\times N_{\text{ENTRIES}}\times N_{\text{TRKS}}. \end{array}$$

The size of a pattern can be used to determine how much time was spent on it in total.

(7) $$\begin{array}{c} T_{\text{TOTAL}}=5\times \left(N_{\text{TRKS}}-7\right)\times \left(T_{\text{SNT}}+T_{\text{OVRHD}}\right)+T_{\text{BIAS}}\times N_{\text{ENTRIES}}\times \sqrt{\text{S}.} \end{array}$$

They apply to any CMPR network configuration with a pattern size greater than unity. In other words, the total time is proportional to the square root of the pattern size. The number of GNs in each position has nothing to do with the length of the learning cycle. As a result, the scheme can support large pattern sizes while only slightly increasing total time.

### 1.3. CMPR Recognizes Patterns

Object recognition uses S&I and GN arrays. The core node receives the pattern and command from the GN arrays. Default index number is determined by the index with the highest percentage of occurrences. If one or more outer tracks cannot generate an index, S&I will keep track of which GNs were voted on.

### 1.4. Genetic Algorithm for the Optimization Process

GAs are an evolutionary algorithm subtype. They are called “adaptive heuristic search algorithms.” Based on natural selection and genetic principles. These are programmes that conduct intelligent random searches, guided by historical data. They are frequently used in high-quality SEO and optimization.

Adaptable species will survive, reproduce, and pass on to the next generation. To solve a problem, they simulate “survival of the fittest” among successive generations. Each generation's members represent a solution and a search space. Characters, integers, floats, and bits represent each person. A chromosome: genetic algorithms analyse population chromosomes. Individuals compete for resources and mates. The most successful (fit) individuals mate to produce the most offspring. Occasionally, due to gene inheritance, parents produce offspring who outperform both parents. As a result, each generation adapts more to its environment.

The search space maintains distinct populations. Each person in the search space represents a solution. Each person has a finite-length component vector (similar to a chromosome). Genes are like these variables. As a result, each chromosome contains many genes (variable components). It measures a person's ability to “compete.” The fittest candidates are preferred. The GAs track individuals' fitness. Higher fitness individuals have a better chance of reproducing than lower fitness individuals. The fittest individuals are chosen to mate and have superior offspring by combining their chromosomes. This is necessary to maintain population stability. Because the elderly population is shrinking, some individuals die and are replaced by newcomers, giving rise to a new generation. Less appropriate solutions will be phased out as more appropriate ones emerge. Environmentally, each generation inherits more “better genes” (solution). As a result, each generation develops better “partial solutions” than the previous one. Convergence occurs when a population's offspring are genetically identical. According to the algorithm, the problem has been solved. Using the operators, the algorithm evolves generation iteratively after initialization. (1) The selection operator's goal is to prioritise fit individuals who will pass on their genes to future generations. (2) The crossover operator represents individual mating. The crossover sites are chosen at random, as are the two individuals. Genes are exchanged at these crossover points, resulting in the birth of a new individual (offspring). (3) Mutation Operator: the idea is to randomly insert genes into offspring to maintain population diversity and prevent premature convergence.

The full algorithm is as follows: (1) Assemble a random population. (2) Determine the population's fitness. (3) Keep going until you reach a point of convergence.

It is necessary to select parents from the population, cross-pollinate the new population, generate mutants, and assess the new population's fitness. The goal is to build a target string from a random string of similar length. These are the characters in chromosome/solution/individual. The fitness score shows how many characters in an index differ from the target string.

### 1.5. Cellular Microscopic Pattern Recognizer (OCMPR) for WSN

(8) $$\begin{array}{c} \text{FP}=\frac{F_{i}}{\sum_{i=1}^{n=6}F_{i}}, \end{array}$$

where FP is fitness probability and *F*_*i*_ is fitness value which is used for the optimization.

This optimization procedure using GA optimizes the parameter of *SI*_*k*_ and *P*_*k*_.

(9) $$\begin{array}{c} {ON}_{k}=\left\{\begin{array}{cc} {SI}_{k}+1, & \text{if no match found}\\ P_{k}, & \text{if a match found} \end{array}\right\},\\ {ON}_{k}=\left\{\begin{array}{cc} 0, & \text{if no match found}\\ P_{k}, & \text{if a match found} \end{array}\right\},\\ ON_{\text{TRKS}}=\left\lceil \sqrt{a}\right\rceil ,\\ {ON}_{\text{PAD}}={\left(N_{\text{TKRS}}\right)}^{2}-a,\\ ON\left(a\right)=v.{\left(\left\lceil \sqrt{a}\right\rceil \right)}^{2},\\ {OT}_{1}=2\times \left(ON_{\text{TRKS}}-1\right)\times \left({OT}_{\text{SNT}}+OT_{\text{OVRHD}}\right). \end{array}$$

*OT*_1_ is excluded from the calculation since there are no nearby nodes at the core node. An array's size affects how long it takes to find a match. Computation time is equal to the greatest single-node computation time for all tracks because all nodes compute simultaneously. Not nodes, but track count determines overall time.

(10) $$\begin{array}{c} {OT}_{2}=OT_{\text{BIAS}}\times ON_{\text{ENTRIES}}\times ON_{\text{TRKS}}. \end{array}$$

This time depends on how frequently nodes report to their inner nodes. Each node has three messages. Two nodes can communicate if assigned. In and out tracks are excluded. Each node sends a message to the outside track. It is all asynchronous.

(11) $$\begin{array}{c} {OT}_{3}=\left(3\times \left({ON}_{\text{TRKS}}-2\right)+1\right)\times \left(OT_{\text{SNT}}+OT_{\text{OVRHD}}\right). \end{array}$$

The sum of the three times *OT*_1_, *OT*_2_, and *OT*_3_ equals the overall learning and recall cycle. As a result, you can calculate the total time required to complete the task as follows:

(12) $$\begin{array}{c} {OT}_{\text{TOTAL}}=5\times \left({ON}_{\text{TRKS}}-7\right)\times \left(OT_{\text{SNT}}+{OT}_{\text{OVRHD}}\right)+{OT}_{\text{BIAS}}\times ON_{\text{ENTRIES}}\times ON_{\text{TRKS}}. \end{array}$$

The size of a pattern can be used to estimate the amount of time spent on it in total.

(13) $$\begin{array}{c} OT_{\text{TOTAL}}=5\times \left({ON}_{\text{TRKS}}-7\right)\times \left(OT_{\text{SNT}}+OT_{\text{OVRHD}}\right)+{OT}_{\text{BIAS}}\times ON_{\text{ENTRIES}}\times \sqrt{S}. \end{array}$$

These relationships apply to any CMPR network with a *S*≥4. The square root of the number of associated positions determines pattern size. The number of GNs in each position has no relation to the cycle length.

## 2. Results and Discussion

We ran three test series on the CMPR. Initially, we looked for crosstalk. To test the scheme's accuracy, we used bitmap image recognition. First, the CMPR was cross-tested. Two or more memorized patterns are recognize as one. In this test, a CMPR network identified 9-bit binary patterns. When using the CMPR as an identifier network, no subpattern combinations are recalled, and no fault-tolerance features are used. There were 512 different patterns. Then, it saved 100 random patterns. It also gave it all 512 recall patterns. After 100 tests, the CMPR only remembered memorised patterns. Our goal was to memorise two distinct patterns that produce subpatterns of initially memorising patterns. This eliminates crosstalk.  Table 1 shows the randomly distorted patterns per memorised between CMPR Detection System and accuracy using binary bitmap image patterns.

Figure 3 shows CMPR Detection System-accuracy in percentage between randomly distorted patterns per memorised.  Table 2 shows the comparison of CMPR average fitness value and GACMPR average fitness value (proposed) using maximum number of generation. As part of the second series test, we memorized the letters “A,” “I,” “J,” “S,” “X,” and “Z.” These letters have no common pattern. So each image was distorted by 1 to 15 bits.  Figure 4 shows distorted stored pattern recall results. Result response rate for each network: in this case, CMPR can detect warped patterns. The CMPR network can recognise A, I, J, and S patterns in 13-bit distortion (36.11 percent). The CMPR network's recall accuracy average recall accuracy of CMPR and HGN: the CMPR is a smaller network with equivalent recall accuracy. The HGN needs 648 nodes to represent 35-length binary patterns using CMPR. A 7 × 5 binary bitmap image pattern was used to model each letter in the third test series. In binary, these letters have similar edges. On each stored pattern, we applied low (5%), medium (11%), and high (11%) distortion. Six figures show average accuracy ratios for 100 randomly deviated patterns. It has a smaller network size (42.86%) but similar recognition accuracy (DHGN).

Figures 5 and 6 show this. We employed the autonomous GA robot steering approach from [11] to test its performance. This method was chosen for its flexibility. Alternatively, any alternative GA-based robot guidance method can be employed. The GA has 0.033 mutation rate, 0.6 crossover rate, and 100 population size. We limit generations at 400 to speed up GA search. This was done to help the GA find optimal training binary map solutions. [11]'s fitness function considers travel length, turns, and collisions. Instead of 0-10, we utilised fitness. The best option is always the best. A 100 × 100 map solution has 102 integer numbers that help a robot navigate. It has 2 transitions.

That is how we compared our GA-AM scheme to the autonomous GA's S&I received the solutions and stored them with the maps. This test dataset was performed eight times, with each run having a distinct maximum generation limit. A total of 100 generations were available for each run time (for both schemes). Setting the maximum generation count allows us to gauge our technique's efficiency. To assure accuracy, both systems employed the same pseudorandom number generator.  Figure 6 compares the two techniques' average fitness and generation values. As shown in Figure 6, the suggested combined GA technique outperforms autonomous GA. Also, a 250-generation mixed GA is preferred over a 400-generation autonomous GA. To solve the 500 test maps, the autonomous GA needed 200000 generations. To discover the best solution for a set of maps, the suggested method requires 127,000 generations (including training). This will eliminate 73000 generations (36.5 percent). The statistics suggest that using CWPR to implant a single solution enhances typical GA performance. The system helps a robot navigate a problem space faster by avoiding obstacles.

The suggested method uses network elements to recognise patterns in a single learning cycle. It also employs fewer nodes than other methods. It also handles noisy patterns, making it excellent for WSN.

## 3. Conclusion

Recognize patterns associated with events to perform event detection. WSN pattern recognition is resource sensitive to computation complexity, iteration count, and node training requirements. Computer-based machine learning is typically iterative. WSN's parallel distributed processing capabilities simplify computations for energy conservation and speed up recognition. The method combines the CMPR with a well-known optimization technique (the genetic algorithm). With limited resources, a WSN's mission-critical applications require this methodology. As a result of the distributed computations and loosely coupled communication, this scheme provides global and rapid recognition while reducing computational constraints. The results demonstrate the proposed scheme's versatility.

## Figures and Tables

**Figure 1:** The input pattern ABBA is responded to and stored by a GN array (4 nodes).

**Figure 2:** Cell GN architecture with two pattern sizes to choose from. (a) To determine a size pattern, sensor nodes were positioned throughout the field of interest. (b) Internode communication in real time. (c) Inner track reporting. Two GN sites per track are separated from their inner GNs by light blue (dotted) arrows. The solid black arrows show how GNs connect to inner track GNs.

**Figure 3:** CMPR Detection System-accuracy in percentage.

**Figure 4:** Comparison on accuracy-CMPR vs. HGN vs. DHGN.

**Figure 5:** CMPR vs. GACMPR schemes-performance.

**Figure 6:** Recognition accuracy results for GACMPR.

**Algorithm 1:** Genetic Algorithm Optimization.

**Table 1:** CMPR Detection System-accuracy in percentage (randomly distorted patterns per memorised).

Binary bitmap image patterns				
A	E	F	K	T
95.34	78.45	63.45	57.89	36.87
94.56	79.63	61.11	54.34	45.74
86.75	74.70	53.21	53.67	32.77
76.88	78.34	51.84	51.78	39.62
82.92	76.59	55.38	50.63	32.64
88.67	62.56	68.96	41.96	31.56
86.56	54.35	45.96	40.32	30.72
78.96	71.34	44.99	39.29	29.43
76.54	70.82	45.98	39.98	30.75
79.65	52.87	48.89	38.43	30.86
76.34	54.89	67.66	33.28	30.22
75.23	68.89	44.78	32.94	29.45
74.56	53.98	34.54	33.32	34.53
76.89	59.76	36.98	32.90	37.76
74.67	63.66	45.53	30.33	34.93

**Table 2:** CMPR vs. GACMPR comparison.

Maximum number of generation	CMPR average fitness value	GACMPR average fitness value (proposed)
50	1.8	7.4
100	7.6	8.1
150	7.9	8.4
200	8.2	8.52
250	8.4	8.7
300	8.5	8.8
350	8.6	8.9
400	8.7	9

## Data Availability

The data used to support the findings of this study are included within the article.
